# Circ_001042 Inhibits TGF-*β*1/P38 MAPK Signaling Axis-Mediated Epithelial-Mesenchymal Transition and Metastasis in Lung Adenocarcinoma

This article has been retracted.

**DOI:** 10.1155/2022/7890490

**Published:** 2022-08-04

**Authors:** Lixia Zhou, Wenxian Chen, Hang Yang, Jiaqin Liu, Hui Meng

**Affiliations:** ^1^Department of Oncology, The Fifth Affiliated (Zhuhai) Hospital of Zunyi Medical University, Zhuhai, Guangdong 519100, China; ^2^Department of Thoracic Surgery, The Fifth Affiliated (Zhuhai) Hospital of Zunyi Medical University. Zhuhai, Guangdong 519100, China

## Abstract

**Objective:**

To explore the role and molecular mechanism of circ_001042 in lung adenocarcinoma (LUAD).

**Methods:**

The expression level of circ_001042 and linear RNA MRPS35 in cells and clinical tissues was detected by real-time PCR (qRT-PCR). The expression of circ_001042 and transforming growth factor *β*1 (TGF-*β*1) in LUAD cells was elevated by the respective transfection of overexpression vectors OE-circ_001042 and TGF-*β*1; MTT and transwell assays were applied to test the proliferation, migration, and invasion abilities of cells, respectively. The E-cadherin expression level in the cells was assessed by immunofluorescence staining, and western blot was utilized to determine the expression level of epithelial-mesenchymal transition (EMT) and TGF-*β*1/P38 MAPK signaling axis-related proteins in the cells.

**Results:**

Circ_001042 was significantly downregulated in LUAD tissues and cells, and high circ_001042 expression could inhibit the proliferation, invasion, and migration of LUAD cells. In addition, circ_001042 also inhibited the EMT process (the E-cadherin level was upregulated; and the levels of N-cadherin, vimentin, and Snail were downregulated) and TGF-*β*1/P38 MAPK signaling axis activity in LUAD cells. Moreover, circ_001042 could suppress the promotion of TGF-*β*1 on the proliferation, invasion, migration, and EMT process of LUAD cells and the activation of TGF-*β*1/P38 MAPK signaling axis.

**Conclusion:**

By inhibiting TGF-*β*1, circ_001042 not only suppresses the proliferation, migration, invasion, and EMT of LUAD but also inhibits the activation of TGF-*β*1/P38 MAPK signaling axis. Therefore, circ_001042 can act as a potential target for early diagnosis and targeted therapy of LUAD.

## 1. Introduction

The International Agency for Research on Cancer reveals that lung cancer (LC) is the leading cause of cancer death worldwide, and approximately 1.8 million people die of LC each year; besides, LC (11.4%) is also the second most common cancer after breast cancer [1]. In recent years, due to the pollution of living environment, the increasing number of smokers, and the smoking tendency in young people, the incidence of LC is growing year by year and the prognosis is very poor [2, 3]. What's worse, LC is diagnosed at an advanced stage in about 85% of patients, which may be one of the main reasons behind the high mortality rate of LC [2, 3]. Non-small cell lung cancer (NSCLC) accounts for about 85% of the total cases of all LCs. NSCLC principally includes lung adenocarcinoma (LUAD), lung squamous cell carcinoma (LUSC), and large cell carcinoma [4]. LUAD is a common type of NSCLC; due to the abundance of blood vessels in the adenoma, the rapid proliferation of tumor cells, and early tumor metastasis, LUAD is also a type of LC with the worst prognosis. Despite significant progress in the treatment, the 5-year survival rate of patients with LUAD is still low; owing to its susceptibility to malignant metastasis, high recurrence rates after treatment and an advanced stage in most of patients have been diagnosed [5, 6]. Consequently, there is an urgent need to find sensitive and effective diagnostic markers for early LUAD and gain insights into the molecular mechanism of LUAD.

MAPK, a member of protein kinase family, widely exists in cells. As a signal transduction system independent of the second messenger, MAPK can transmit extracellular information to the inside of cells, thus participating in the regulation of cell mitosis, metabolism, programmed death, inflammatory response, and other physiological processes and playing an important role in the immune response to a variety of diseases [7]. It has reported that SPA0355 is a thiourea derivative with antioxidant and anti-inflammatory activities, suppressing activation of the MAPKs pathway to prevent bone loss in mice [8]. P38 MAPK plays an important role in tumor cell invasion and metastasis. Many studies have shown that P38 MAPK signal regulates epithelial-mesenchymal transition (EMT), which is related to tumor invasion and metastasis [9, 10].

Circular RNAs (circRNAs) belong to closed noncoding RNAs and can stably present in mammals [11]. Characterized by high stability, conservation, and specific expression, circRNA does not have a 5′ terminal cap and 3′ terminal tail and can be composed of both exon splicing and intron splicing [12]. In recent years, a number of studies have confirmed that circRNAs participate in a variety of human disease progression by adsorbing microRNAs, regulating the function of target microRNAs, and regulating gene expression at the post-transcriptional level [13]. And the human disease progressions involved by circRNAs include colon cancer [14], ovarian cancer [15], gastric cancer [16], esophageal cancer [17], glioma [18], and LUAD [19]. From the above, circRNAs can be seen as one of the potential targets for cancer diagnosis and treatment. Circ_001042 is a newly discovered circRNA with a total length of 147 bp, and there is no detailed study on circ_001042 currently. Circ_001042 is located in Chromosome 2 and is an intergenic circRNA. Only a bioinformatics study [20] by Li et al. revealed the close correlation between circ_001042 and multiple anorectal malformation (ARM)-related signaling pathways. And the function and mechanism of circ_001042 in diseases such as cancer are unknown. Therefore, in this study, circ_001042 expression in LUAD tissues and cells of patients was detected. Specifically, through a series of cell biology and molecular biology experiments, we explored the role and possible mechanism of circ_001042 in malignant biological behaviors such as proliferation, migration, invasion, and the EMT process of LUAD cells. And all the above in this paper were to excavate new biomarkers for the diagnosis and treatment of LUAD.

## 2. Materials and Methods

### 2.1. Tissue Specimens

We collected 10 tumor tissues (LUAD group) and 10 adjacent normal histological tissues (normal group) from LUAD patients who underwent surgery in The Fifth Affiliated (Zhuhai) Hospital of Zunyi Medical University, 10 tumor tissues from metastatic LUAD patients (metastasis), and 10 tumor tissues from nonmetastatic LUAD patients (nonmetastasis). This study was approved by the Ethics Committee of The Fifth Affiliated (Zhuhai) Hospital of Zunyi Medical University (No.2022ZH061), and all experiments were carried out in accordance with the approved guidelines. All patients signed informed consent.

### 2.2. Cell Culture and Transfection

Human normal lung epithelial cells (BEAS-2B) and LUAD cells A549 and H460 were purchased from the National Collection of Authenticated Cell Cultures. The above cells were cultured in RPMI-1640 medium supplemented with 10% fetal bovine serum (FBS; Gibco, USA) and 1% penicillin streptomycin (Gibco, USA) in a cell incubator at 37°C, 5% CO_2_, and 95% humidity. Plasma cells were cultured to the logarithmic growth phase, then digested, and passaged.

A549 and H460 cells in the logarithmic growth phase were collected, resuspended, and then seeded in a 6-well plate. When cell confluence reached 80%, transfection was performed. Specifically, the transfection of A549 cells was divided into vector group, OE-circ_001042 group, control group, transforming growth factor *β*1 (TGF-*β*1) group, TGF-*β*1 + vector group, and TGF-*β*1 + circ_001042 group. The transfection of H460 cells was divided into vector group and OE-circ_001042 group. The foresaid vectors were transfected into the corresponding cells based on the transfection instructions of lipo2000 reagent, and after 48 h, transfected cells were collected.

### 2.3. Real-Time PCR

Total RNA was extracted from the collected cells with a total RNA extraction kit (Beyotime, China). And the extracted RNA was stored at −80°C, followed by reverse transcription to synthesize cDNA according to the instructions of the reverse transcription PCR kit (Takara, Japan). The synthesized cDNA was utilized to determine the expression of circ_001042 and TGF-*β*1 based on the instructions of the real-time PCR kit (Takara, Japan). Data analysis was performed with the 2^−ΔΔCt^ method, and the relative expression level of the target gene was calculated using *β*-actin as an internal control. The primers are as follows: circ_001042: F: 5′-GACTTCGCAGGCGTAGACTT-3′, R: 5′-CCCGTCACAAAGAGCTTCAA-3′; TGF-*β*1: F: 5′-CCACCTGCAAGACCATCGAC-3′, R: 5′-CTGGCGAGCCTTAGTTTGGAC-3′; MRPS35: F: 5′-CCACCAAGAAGAAAGGCACTAC-3′, R: 5′-GTGCTGCAACTGGGTAAACAC-3′; *β*-actin: F: 5′-GGCTGTATTCCCCTCCATCG-3′, R: 5′-CCAGTTGGTAACAATGCCATGT-3′.

### 2.4. MTT Assay

The cell specimens were collected, and the cell concentration was adjusted to 3 × 10^4^ cells/ml. Then, 100 *μ*l of cells were seeded in a 96-well plate with 6 replicates for each group. The cells were cultured in a cell incubator until the cell adhesion was presented. Next, the cell proliferation was determined at 0 h and 24 h after adherence according to the instructions of the MTT kit (Beyotime, China). Briefly speaking, cell culture was continued for 4 h after adding 20 *μ*l of MTT solution (5 mg/ml) to the wells of the plate. Later, the supernatant was removed, and 100 *μ*l of formazan lysis solution was added to each well for subsequent culture. And the cell culture was discontinued when formazan crystals were all dissolved. Finally, a microplate reader was employed to determine the absorbance value at 570 nm.

### 2.5. Transwell Assay

Firstly, 100 *μ*l of Matrigel diluted with serum-free medium was added into the upper chamber of transwell, and the chamber was placed in a cell incubator at 37°C for 3–5 h to convert diluted Matrigel into solid state. The following procedures were the same as those for the migration test. To be specific, the cells were collected and resuspended with serum-free medium. After the concentration was adjusted to 5 × 10^5^ cells/ml, more than 100 *μ*l of cell suspension was added into the upper chamber, and 600 *μ*l of medium containing 20% FBS into the lower chamber. After 18–24 h of culture, the cells and Matrigel that did not pass through the membrane in the upper chamber were carefully wiped off with a cotton swab. Then, 4% paraformaldehyde was added for cell fixation, and a crystal violet solution was adopted for cell staining. After being dried, the cells were photographed under a microscope and counted statistically.

### 2.6. Immunofluorescence Staining

After the cell culture medium was removed, the LUAD cells in each well were washed with PBS (5 min × 3 times), followed by fixation with 3.65% methanol, penetration with 0.2% Triton X-100, and blocking with 5% BSA. After that, cells were incubated overnight at 4°C with addition of E-cadherin antibody (CST, USA). After washing the cells with PBS (5 min × 3 times), immunofluorescence secondary antibody (CST, USA) was added for another incubation in the dark for 2 h. Again, the cells were washed with PBS (5 min × 3 times), then 20 L/L DAPI solution was dripped, and the coverslip was covered to avoid the generation of bubbles. After 5 min, observation and photographs of the treated cells under a fluorescence microscope were performed.

### 2.7. Western Blot

LUAD cells from each group were collected and lysed on ice for 20 min by adding RIPA lysate (Solarbio, China) followed by sonication of cells in an ice bath. After centrifugation at 10,000 rpm and 4°C, total cell protein in the supernatant was collected, and the protein concentration was detected according to the instructions of the BCA kit (Beyotime, China). Later, 30 *μ*g of protein was separated by SDS-PAGE (sodium dodecyl sulfate-polyacrylamide gel electrophoresis), and then the target protein was transferred to a PVDF membrane. Subsequently, 5% skimmed milk powder was added for 2 h blocking, and diluted primary antibody (CST, USA) was added for incubation overnight at 4°C. After being washed three times with TBST, the membrane was incubated with diluted secondary antibody (Zhongshan Golden Bridge Biotechnology Co., Ltd., China) at ambient temperature for 1 h. After adding ECL chemiluminescence solution, the protein was developed in a gel imager and then was photographed and archived. Finally, the gray level of the bands was calculated using Image-Pro Plus and the protein level was analyzed with *β*-actin as an internal control.

### 2.8. Statistical Analysis

All results were expressed as mean ± standard deviation (SD), and SPSS 21.0 software was employed for statistical analysis. A *T*-test was utilized for comparison between two groups, and one-way analysis of variance for comparison among multiple groups. *P* < 0.05 was considered as a statistically significant difference.

## 3. Results

### 3.1. Downregulation of Circ_001042 in LUAD Tissues and Cells

Firstly, circ_001042 expression in clinical tissues (LUAD tissues and normal tissues) was examined. And the examination outcomes revealed that circ_001042 expression in LUAD tissues was much lower than that in corresponding normal tissues (*P* < 0.01, Figure 1(a)). And circ_001042 expression in the metastasis group was notably lower than that in the nonmetastasis group (*P* < 0.01, Figure 1(b)). Also, the circ_001042 expression level in LUAD cells A549 and H460 was greatly lowered down compared with that in normal lung epithelial cells BEAS-2B (*P* < 0.01, Figure 1(c)). Besides, after RNase R treatment, circ_001042 expression was evidently higher than linear RNA MRPS35 expression in A549 and H460 cells (*P* < 0.01, Figure 1(d) and 1(e).

### 3.2. Circ_001042 Inhibits the Proliferation, Migration, and Invasion of LUAD Cells

To clarify the function of circ_001042 in LUAD, circ_001042 expression in A549 and H460 cells was increased by transfection with OE-circ_001042 (Figure 2(a) and 2(b)). Subsequently, the effect of circ_001042 overexpression on the proliferation, migration, and invasion of LUAD cells was tested by MTT and transwell, respectively. The results showed that the proliferation rate, migration, and invasion abilities of A549 and H460 cells in the OE-circ_001042 group were obviously lower than those in the vector group (*P* < 0.01, Figure 2(c)–2(g)). The above suggested that circ_001042 inhibited the proliferation, migration, and invasion of LUAD cells.

### 3.3. Circ_001042 Inhibits Epithelial-Mesenchymal Transition (EMT) Progression in LUAD Cells

The effect of circ_001042 on the EMT process of LUAD cells was assessed by immunofluorescence staining and western blot. And immunofluorescence results demonstrated that the fluorescence staining intensity of E-cadherin in A549 and H460 cells from the OE-circ_001042 group was notably enhanced compared with the vector group (Figure 3(a)). In addition, the protein expression level of vimentin, N-cadherin, and Snail in A549 and H460 cells in the OE-circ_001042 group was markedly lower than that in LUAD cells in the vector group (*P* < 0.01, Figure 3(b) and 3(c)). The above indicated that circ_001042 inhibited EMT progression in LUAD cells.

### 3.4. Circ_001042 Inhibits TGF-*β*1/P38 MAPK Signaling Axis in LUAD Cells

It is reported that TGF-*β*1 can induce EMT progression in various tumor cells such as ovarian, gastric, and breast cancers [21–23]. To determine whether high circ_001042 expression inhibited EMT progression in LUAD cells through a TGF-*β*1-dependent signaling pathway, we examined the TGF-*β*1-dependent signaling pathway by western blot. The results presented that overexpression of circ_001042 inhibited the expression of TGF-*β*1 as well as the phosphorylation of Smad3 and P38 and significantly reduced the ratios of p-Smad3/Smad3 and p-P38/P38 (Figure 4(a) and 4(b)). Therefore, we speculated that circ_001042 inhibited EMT progression by decreasing the activity of TGF-*β*1/P38 MAPK signaling pathway in LUAD cells.

### 3.5. Circ_001042 Inhibits A549 Cell Proliferation, Invasion, Migration, and EMT Progression by Downregulating TGF-*β*1

To further verify that circ_001042 played a cancer-inhibiting role by regulating TGF-*β*1, the expression of TGF-*β*1 was overexpressed by transfection. And according to the cell function analysis in each group, compared with the control group, the TGF-*β*1 group exhibited a noticeable increase in the proliferation rate, invasion, and migration abilities of cells, a remarkable decrease in the E-cadherin fluorescence intensity, and a marked rise on the protein expression level of vimentin, N-cadherin, and Snail (*P* < 0.01); furthermore, the proliferation rate, invasion, and migration abilities of A549 cells in the TGF-*β*1 + circ_001042 group were greatly declined compared with those in the TGF-*β*1 + vector group; the fluorescence intensity level of E-cadherin in the cells was significantly increased; and the protein expression level of vimentin, N-cadherin, and Snail was notably decreased (*P* < 0.01); however, there was no significant difference in the TGF-*β*1 group and TGF-*β*1 + vector group (*P* > 0.05) (Figure 5(a)–5(g)). All in all, overexpression of TGF-*β*1 could significantly promote the proliferation, migration, invasion, and EMT process of A549 cells, while overexpression of circ_001042 could reverse the promoting effect of TGF-*β*1 on the proliferation, invasion, migration, and EMT process of A549 cells.

### 3.6. Circ_001042 Inhibits TGF-*β*1/P38 MAPK Signaling Axis Activated by TGF-*β*1

The effect of circ_001042 on the activity of TGF-*β*1/P38 MAPK signaling axis activated by TGF-*β*1 in A549 cells was further verified. As results shown, compared with the control group, the TGF-*β*1 group presented a marked increase in the protein expression level of TGF-*β*1, p-Smad3, and p-P38 as well as the ratios of p-Smad3/Smad3 and p-P38/P38 in A549 cells. However, compared with the TGF-*β*1 + vector group, a noticeable reduction could be observed in the protein expression level of TGF-*β*1, p-Smad3, and p-P38 and the ratios of p-Smad3/Smad3 and p-P38/P38 in A549 cells in the TGF-*β*1 + circ_001042 group; in addition, there were no significant differences between TGF-*β*1 and TGF-*β*1 + vector groups (*P* > 0.05) (Figure 6(a) and 6(b)). In summary, TGF-*β*1 could highly activate the TGF-*β*1/P38 MAPK signaling axis, while overexpression of circ_001042 could greatly inhibit TGF-*β*1/P38 MAPK signaling axis activity induced by TGF-*β*1.

## 4. Discussion

LC is one of the main causes behind reduced survival in cancer patients, with high incidence and mortality [24]. What's worse, the metastasis and poor prognosis of LC make its treatment face great challenges [25]. At present, there is no effective diagnostic tool to distinguish LUAD patients at early and advanced stage. With the development of high-throughput sequencing technology, more and more studies have reported a close association of the abnormal expression of noncoding RNAs with the occurrence and malignant behavior of a variety of cancers [19]. As an emerging molecule, circRNAs have received increasing attention in recent years. Some studies have revealed that abnormal expression of circRNA plays an important role in the occurrence and progression of a variety of tumors. Circ_001042 is a newly discovered circRNA whose function in diseases such as cancers is unknown. In this study, qRT-PCR results showed that the circ_001042 expression level was remarkably downregulated in LUAD tissues and cells, and circ_001042 expression was much lower in metastatic LUAD patients than that in nonmetastatic LUAD patients; besides, overexpression of circ_001042 inhibited the proliferation, invasion, and migration of LUAD cells. The above findings in this study suggested that circ_001042 played a cancer-inhibiting role in LUAD.

Studies have shown that EMT is considered to be one of the important mechanisms of malignant process, invasion and metastasis of tumor cells. Specifically, EMT is principally manifested as the loss in epithelial cell morphology, cell polarity, tight junctions, the decrease in intercellular adhesion, and the transformation to mesenchymal cell morphology with invasive and metastatic ability [26]. In fact, EMT is very critical in the process of tumor invasion and metastasis. It is reported that E-cadherin will transform into N-cadherin during EMT, so E-cadherin expression, as an epithelial cell marker, is downregulated, while N-cadherin, vimentin, and Snail, as mesenchymal cell markers, are upregulated [27]; and the expression change of the above proteins is one of the basic markers of EMT development [28]. Moreover, related research revealed a worse prognosis in tumor patients with high expression of vimentin and Snail [29,30]. In this study, overexpression of circ_001042 greatly increased the E-cadherin expression level and decreased the protein expression level of vimentin, N-cadherin, and Snail, indicating that high expression of circ_001042 inhibited the EMT process of LUAD cells. And previous studies have also reported that a series of circRNAs such as circ_0092367 and circ_0043265 can suppress cancers by inhibiting the EMT process [31,32].

Research projects have reported that EMT can be triggered by multiple signaling molecules. For example, TGF-*β* regulates the EMT process mainly through the Smad and non-Smad pathways. Specifically, TGF-*β* extracellularly binds to TGF-*β*RII to activate TGF-*β*RI firstly; then the activated TGF-*β*RI phosphorylates Smad2/3; and the phosphorylated Smad2/3 binds to Smad4 to become a complex; finally, the complex enters the nucleus to regulate corresponding target gene transcription together with other transcription factors and to play a significant role in cell proliferation, differentiation, apoptosis, and migration [33,34]. The MAPK signaling pathway, namely, mitogen-activated protein kinase signaling pathway, is an intracellular signaling molecule of the EMT process and a common path for cell membrane-to-nuclear responses caused by extracellular stimulation signals. As studies shown, MAPK can activate NF-kB; and the activated NF-kB can induce EMT in cells by promoting cell proliferation and reducing the expression of E-cadherin and keratin [35]. Some papers have revealed that TGF-*β*1 can induce EMT in LUAD cells; and the induced LUAD cells present a morphology transformation from an epithelial cell phenotype to a mesenchymal cell phenotype, a downregulation in E-cadherin expression, an upregulation in N-cadherin and vimentin expression, and an enhancement in invasion and migration abilities [36]. In this study, overexpression of circ_001042 significantly reduced the protein expression level of TGF-*β*1, p-Smad3, and p-P38, greatly declined the ratios of p-Smad3/Smad3 and p-P38/P38, and then inhibited the activation of the TGF-*β*1/P38 MAPK signaling axis in LUAD cells. Additionally, circ_001042 inhibited LUAD cell proliferation, invasion, migration, and EMT progression by inhibiting TGF-*β*1-activated TGF-*β*1/P38 MAPK signaling axis.

In this study, only the inhibitory effect of circ_001042 on the malignant behavior of LUAD was demonstrated by cell experiments, and only the TGF-*β*1/P38 MAPK signaling axis was measured. Also, neither validations of *in vivo* experiments in animals nor explorations of other potential mechanisms were performed, and the specific regulatory mechanism of TGF-*β*1 to circ_001042 also kept unclear. The lack of or downregulation of circ_001042 in LUAD patients may indicate that the prognosis of patients is poor, and there is a risk of tumor metastasis. Circ_001042 is expected to be a potential biomarker and therapeutic target for predicting metastasis of LUAD. CircRNAs mainly function as “sponges” of microRNAs through competitive endogenous RNA (ceRNA) networks. And bioinformatics studies of Li et al. have indicated that circ_001042 not only is associated with miR-92a-1-5p but also may act as ceRNA to regulate the progression of ARM [20]. We speculated that circ_001042 may exert target gene regulation effects by sponging a miRNA and then to inhibit the progression of LUAD. Therefore, more experiments need to be carried out for further exploration.

## 5. Conclusions

To summarize, circ_001042 is downregulated in LUAD tissues and cells, and circ_001042 overexpression can inhibit the proliferation, invasion, migration, and EMT process of LUAD cells. In addition, overexpression of circ_001042 can play a role in cancer inhibition by reversing the TGF-*β*1-induced malignant behavior of LUAD cells and activity increase in the TGF-*β*1/P38 MAPK signaling axis. In conclusion, circ_001042 has potential as a marker for early diagnosis and targeted therapy of LUAD.

## Figures and Tables

**Figure 1:** Downregulation of circ_001042 in LUAD tissues and cells. A–C qRT-PCR to determine the circ_001042 expression level in the LUAD/normal groups (a), metastasis/nonmetastasis groups (b), and BEAS-2B, A549, and H460 cells (c), ^*∗∗*^*P* < 0.01 vs BEAS-2B. (d) and (e) qRT-PCR was employed to determine the expression level of circ_001042 and linear RNA MRPS35 in A549 and H460 cells, respectively, ^*∗∗*^*P* < 0.01.

**Figure 2:** Circ_001042 inhibits the proliferation, migration, and invasion of LUAD cells. A/B qRT-PCR to detect the circ_001042 expression level in A549 (a) and H460 (b) cells in the vector and OE-circ_001042 groups; C/D MTT was used to determine the proliferation rate of A549 (c) and H460 (d) cells in the vector and OE-circ_001042 groups; and E–G transwell was used to check the migration and invasion abilities of A549 and H460 cells in the vector and OE-circ_001042 groups, ^*∗∗*^*P* < 0.01.

**Figure 3:** Circ_001042 inhibits epithelial-mesenchymal transition progression in LUAD cells. (a) Immunofluorescence staining to assess the expression of E-cadherin in A549 and H460 cells in the vector and OE-circ_001042 groups; and (b) and (c) western blot to detect the protein expression level of vimentin, N-cadherin, and Snail in A549 and H460 cells in the vector and OE-circ_001042 groups, ^*∗∗*^*P* < 0.01.

**Figure 4:** Circ_001042 inhibits the TGF-*β*1/P38 MAPK signaling axis in LUAD cells. (a) and (b) Western blot was utilized to determine the protein expression level of TGF-*β*1, p-Smad3, Smad3, p-P38, and P38 in A549 and H460 cells in the vector group and OE-circ_001042 groups, ^*∗∗*^*P* < 0.01 vs vector.

**Figure 5:** Circ_001042 inhibited the proliferation, invasion, migration, and EMT process of A549 cells induced by TGF-*β*1. (a) MTT to detect the proliferation rate of A549 cells in each group; B–D transwell to test the invasion and migration abilities of A549 cells in each group; (e) immunofluorescence staining to determine the level of E-cadherin in A549 cells in each group; and F/G western blot to check the protein expression level of vimentin, N-cadherin, and Snail in A549 cells in each group, ^*∗∗*^*P* < 0.01 vs control, ^##^*P* < 0.01 vs TGF-*β*1.

**Figure 6:** Circ_001042 inhibits the TGF-*β*1/P38 MAPK signaling axis activated by TGF-*β*1. (a) and (b) Western blot to detect the protein expression level of TGF-*β*1, p-Smad3, Smad3, p-P38, and P38 in A549 cells of each group, ^*∗∗*^*P* < 0.01 vs control, #*P* > 0.05, and ^##^*P* < 0.01 vs TGF-*β*1.

## Data Availability

The data used to support the findings of this study are available from the corresponding author upon request.
